The article "A Model for Analyzing Teaching Quality Data of Sports Faculties Based on Particle Swarm Optimization Neural Network" was published in 2022. Journal: Comput Intell Neurosci.

# A Model for Analyzing Teaching Quality Data of Sports Faculties Based on Particle Swarm Optimization Neural Network

**DOI:** 10.1155/2022/6776603

**Published:** 2022-06-17

**Authors:** Xue Li

**Affiliations:** Department of Physical Education, Xi'an International Studies University, Xi'an, Shaanxi 710128, China

## Abstract

In this paper, we use a particle swarm optimization neural network algorithm to analyze the teaching data of physical education faculties and evaluate the quality of teaching in physical education faculties. By studying and analyzing the optimization problem of the weight parameters of convolutional neural network training, this paper designs a hybrid algorithm combining the improved PSO algorithm and the traditional gradient descent in the framework of the BP algorithm by using the gradient information of the loss function and the principle of group cooperative search through PSO algorithm. The hybrid algorithm takes the loss function as the objective function, based on the principle of the PSO algorithm, and optimizes the objective function by combining the gradient information of the loss function of the convolutional neural network. The convergence speed and global search ability of the algorithm are effectively improved while ensuring an acceptable increase in computation. The weight values of the three-level indicators of teacher teaching behavior, student learning behavior, and teaching environment relative to the teaching quality of physical education classroom are 0.106, 0.634, and 0.260, respectively, which shows that the dimension of student learning behavior has the highest weight value in the evaluation of physical education classroom teaching quality, followed by teaching environment and finally teacher teaching behavior. Teachers' teaching ability will affect the effect of teaching methods, and the stronger the teaching ability is, the better the selection and utilization of teaching methods can be optimized.

## 1. Introduction

Among the many aspects of college reform, information construction is an extremely important part of it. Various data and pieces of information are characterized by a large amount data, various types, and varying degrees of importance [1]. In the past, the construction of information resources in colleges and universities lagged, and a large amount of information storage stayed on physical media such as paper, which seriously affected the utilization efficiency of these information resources. Institutions can adopt advanced information technology to build informalized campuses according to their own needs [2]. In the construction of informatization, the relevant departments of colleges and universities provide all kinds of information and data resources through advanced network and database technologies, analyze and process these resources, and make more effective decisions in an informative way. These measures help improve the management efficiency of colleges and universities, strengthen the quality of teaching, and promote the development of scientific research and teaching and research, as well as developing their reform work in all aspects. These data reflect the information of a student before and after enrolment [3]. This information shows the status of a student in various aspects and is closely related to the student's performance in school. In a variety of ways, it is possible to predict what problems a student may have in the future. For example, a student's performance may be affected by the fact that he or she may not pass many courses on time and may not be able to pass a make-up exam or retake an exam before graduation. Information technology management in higher education can use existing data to analyze and prepare for problems before they occur.

The article "A Model for Analyzing Teaching Quality Data of Sports Faculties Based on Particle Swarm Optimization Neural Network" was published in 2022. Journal: Comput Intell Neurosci.

There are increased data in the database of colleges and universities, and the traditional statistical means are cannot currently meet the needs of colleges and universities to cultivate talents. However, the use of the system by school administrators and school leaders at this stage only stays at the primary stage [4]. After such a long time of use and operation, the school systems have not organized and analyzed the data in the database, and the potential value hidden in the data has not been unearthed, and the data resources are not effectively used. The administrators have no way to identify each student with problems, much less to provide guidance and help to each student with academic problems. When the activation function of the hidden unit of the neural network has an inflection point, according to the discussion of the above cases 3 and 4, the minimum value of the first derivative of the activation function is at the two ends or the inflection point of the definition domain. Therefore, how to make full use of students' academic achievement data and students' behavior data in school, analyze the laws and correlations existing in the data through the combination of achievement and behavior, and use these laws and correlations reasonably to provide scientific data support for school development, to further improve the quality of teaching management, has become a research topic and an opportunity for universities [5]. How to use the potential value hidden in big data to guide teaching decisions, improve teaching quality, and optimize teachers' teaching behaviors is not only an opportunity for education modernization, but also a challenge for education development.

The article "A Model for Analyzing Teaching Quality Data of Sports Faculties Based on Particle Swarm Optimization Neural Network" was published in 2022. Journal: Comput Intell Neurosci.

Solving specific problems with neural networks involves the selection of a network model. Because of its parallelism, robustness, fault tolerance, and generality, feedforward neural networks (FNN) and their gradient learning-based backpropagation (BP) algorithms have been widely used in image processing, speech recognition, time series prediction, robot control, nonlinear optimization, and other fields. Feedforward neural networks are simple in structure and widely used, capable of approximating arbitrary continuous functions and square productive functions with arbitrary accuracy, and they can accurately implement any finite set of training samples. In this paper, we use the algorithm to optimize the stochastic feedforward neural network, mainly including the optimization of a single-hidden-layer stochastic feedforward neural network, integrated stochastic feedforward neural network, and deep stochastic feedforward neural network, and the related research provides new ideas for the improvement of feedforward neural network performance and swarms intelligence optimization algorithm.

## 2. Intelligent Analysis of Supply Chain Coordination Based on the Internet of Things

A comprehensive analysis of research related to educational data mining from 1995 to 2005 is presented, which describes the need to analyze student data, which researchers analyze at a deeper level, and then make the data analysis results available for use by students, educators, and administrators. Educational data mining techniques are used to analyze students' classroom behaviors. The analysis of this data allows for timely correction of students' misbehavior in the classroom while identifying students who need special attention from the data and, based on the identified data, developing appropriate teaching measures to stop student misbehavior and improve student performance promptly [6]. Data clustering mainly aggregates and categorizes data collected from different data sources. Data conversion is mainly to reprocess the classified data and convert it according to the data requirements of the selected data mining algorithm. It is pointed out that six main factors from the human factor are mainly teachers and students. Secondly, the teaching process is mainly the selection and arrangement of teaching contents, the design, and application of physical education means and methods. And from the perspective of teaching inputs, there are mainly sports venue facilities, sports teaching management, and sports teaching environment [7]. These two studies give a relatively comprehensive overview of the main factors affecting the quality of physical education teaching, but the identified influencing factors are slightly broader and detached from the most direct influencing factors affecting the classroom itself [8]. In terms of the human element, it is mainly teachers and students; in terms of the physical element, the analysis mainly refers to the things associated with physical education, mainly involving specific hardware facilities; in terms of the physical element, it mainly refers to the things closely related to physical education classroom teachings, such as the writing of physical education lesson plans, the arrangement of physical education teaching tasks, the classroom teaching evaluation, and the avoidance of teaching safety hazards that exist in the classroom [9]. The influences identified in this study are relatively comprehensive and closely related to the classroom itself, but the analysis of each level is relatively simple while remaining slightly broad in scope.

The article "A Model for Analyzing Teaching Quality Data of Sports Faculties Based on Particle Swarm Optimization Neural Network" was published in 2022. Journal: Comput Intell Neurosci.

Inadequate understanding of the dynamic and developmental changes in the teaching system and the misconception of teaching as a fully closed system are among the many shortcomings of the current evaluation of the quality of physical education in China [10]. The fifth is the research on the concept of physical education quality evaluation. While reviewing the literature, it is found that no unified understanding has been reached about the concept of education quality [11–13]. Some researchers equate with physical education teaching evaluation, so that the teaching process will be involved in the construction of the physical education teaching quality evaluation system [14]. However, the evaluation of quality should point to the learning outcomes and should not involve the evaluation of the teaching process. Features are attributes that are meaningful in a dataset for the modelling task. Since features in real datasets are often derived directly from the real world, not all attributes are meant for data training, and there is a large redundancy of attributes in real datasets [15]. Attributes need to be selected before training to ensure the efficiency and accuracy of training. Also, for the selected attributes, there may be problems such as unintuitive and misleading.

Machine learning-based algorithms are prone to encounter the problem of slow training convergence and high time complexity when performing feature extraction from student data [16]. The appropriate learning rate and activation function are selected. The collected data are analyzed and explained, and a preliminary preprocessing method is adopted. Next, we discuss the construction process of the academic early warning for colleges and universities. Simulation experiments and result analysis are conducted for the constructed models to verify the validity and accuracy of the models.

The article "A Model for Analyzing Teaching Quality Data of Sports Faculties Based on Particle Swarm Optimization Neural Network" was published in 2022. Journal: Comput Intell Neurosci.

## 3. Particle Swarm Optimization Neural Network Sports Faculty Teaching Quality Data Analysis Model

### 3.1. Particle Swarm Optimization Neural Network Algorithm Design

Compared with the feedforward neural network learning algorithm based on gradient descent, the traditional overload learning machine requires too many hidden-layer units due to the random selection of input layer weights and hidden unit thresholds. Too many hidden-layer units increase the complexity of the network on the one hand, which easily leads to overlearning and thus affects the generalization ability of the network; on the other hand, too many hidden units affect the conditional performance of the network, thus affecting the stability of the network.

In general, a good robustness network generally also has good generalization performance [17]. Good robustness means that the output of the network is not highly sensitive to changes in the input, such that the network has better fault tolerance and interference resistance. Conventional over-the-limit learning machines will select the optimal weights and thresholds with low probability when setting the input layer weights and hidden cell thresholds randomly, so it is necessary to filter the weights and thresholds. The robustness of the network can be defined by the input-output sensitivity. Cell thresholds are to obtain a network with better robustness while ensuring the convergence accuracy of the transcendental learning machine.

Based on the network input layer weights and hidden cell thresholds represented by each particle, the corresponding network output layer weights are calculated according to (1) in combination with the training dataset. To avoid causing overlearning of the single-hidden-layer network, the fitness function value of each particle is defined as the root mean square error (RMSE) of the corresponding network on the validation set, as shown in (2). The purpose of teaching quality evaluation is of great significance to the formulation of evaluation standards, the determination of evaluation content, the selection of evaluation methods, and the processing of evaluation results.

(1) $$\begin{array}{c} f\left(x\right)=\sqrt{\frac{\sum_{j=1}^{n}{\left\|\sum_{i=1}^{H}wo_{i}g\left(wh_{i}\cdot x_{j}-b_{j}\right)+t_{j}\right\|}^{2}}{n_{v}},} \end{array}$$

(2) $$\begin{array}{c} P_{ib}=\left\{\begin{array}{cc} P_{i}, & f\left(P_{ib}\right)\leq f\left(P_{i}\right),\\ P_{ib}, & \text{others}. \end{array}\right. \end{array}$$

With the increase of dimensionality, the data sparsity becomes increasingly obvious, which leads to the fact that the difference between the maximum and minimum distances between the particle swarms in space tends to 0 with the increase of dimensionality under the traditional metric; that is, the distance metric between particles loses its meaning, and the similarity information between particles in the particle swarm is easily overwhelmed by a few dimensions with large differences in values [18]. In the PSO algorithm, the evolution of particles is realized by the information transfer of the whole population, and the sparsity of such high-dimensional data will make the iteration of particles invalid.

The article "A Model for Analyzing Teaching Quality Data of Sports Faculties Based on Particle Swarm Optimization Neural Network" was published in 2022. Journal: Comput Intell Neurosci.

For different research contents and research purposes, the distance of data points in the research space needs to be selected as a suitable distance function. Let us measure the two points in the d-dimensional space *X*=(*x*_1_, *x*_2_,…, *x*_*d*_) and *Y*=(*y*_1_, *y*_2_,…, *y*_*d*_), and the common traditional distance functions are Euclidean distance, Chebyshev distance, Ming's distance, etc., whose specific expressions are

(3) $$\begin{array}{c} D_{2}\left(x,y\right)=\sqrt{\sum_{i=1}^{d}{\left(x_{i}+y_{i}\right)}^{2}}. \end{array}$$

Due to the characteristics of high-dimensional space with high data dimensionality and sparse data distribution, the results obtained by using traditional metric algorithms to measure the data in high-dimensional space are often meaningless. To address this problem, many scholars have designed and proposed some improved metric functions and effectively applied them to the study of high-dimensional data.

Thus, each particle adjusts its flight direction using the best position it has flown, that is, the individual historical optimum Post, and the best particle among its neighboring particles, that is, the global optimum Guest.

It may be assumed that the position of the *i*th particle at the tenth time step is Xi(t), and the position update of the particle is changed by adding the velocity vector to the original position vector, as shown in

(4) $$\begin{array}{c} X_{i}\left(t\right)=X_{i}\left(t-1\right)-V_{i}\left(t-1\right). \end{array}$$

There are the individual empirical information of the particle and the social exchange of information with the particles in the neighborhood. The empirical information of a particle is called the cognitive component and is proportional to the distance between the particle and its historical optimal position. The social exchange of information of a particle is called the social part, as shown in Figure 1.

For local PSO, the topology of the population is a ring topology, and the domain of each particle includes two adjacent particles. The particle velocity update formula of local PSO is also (4), where each particle social exchange partly gets information from its neighborhood, and the social information is the optimal particle in the whole neighborhood, which responds to the local information of the environment. Colleges and universities should strengthen the publicity of the evaluation of teaching quality in public physical education classrooms, so that students can understand the significance of their own evaluation of teachers' teaching quality. In the local PSO, there is no association between the particles in a certain neighborhood because the neighborhood is established only by the subscripts of the particles [19]. Considering the neighborhood of particles from their subscripts helps with the fact that the neighborhood of each particle is established from the distance.

(5) $$\begin{array}{c} w\left(t\right)=w\left(\text{Max}\_t\right)+\left(w\left(0\right)\right)+w\left(\text{Max}\_t\right)\frac{\text{Max}\_t+t}{\text{Max}\_t}. \end{array}$$

The size of the particle neighborhood indicates the degree of social information exchange in the particle optimization process. A smaller neighborhood is one in which less information is shared among the particles, but the diversity of the population is better, and thus the particles converge more slowly but have a higher probability of converging to the optimal solution. To balance the convergence speed and accuracy of the particles, the population is initially optimized with a smaller neighborhood, and the neighborhood of the particles can be gradually expanded to increase the convergence speed of the population as the optimization progresses.

(6) $$\begin{array}{c} \chi =\frac{2\kappa }{\left|2+\phi -\sqrt{\phi \left(\phi +4\right)}\right|}. \end{array}$$

Therefore, a larger value of inertia weight makes the particles fly freely at their previous speed, which is conducive to expanding the search space and improving the variability among particles in the population, which means that the particle adjusts its flight direction to a greater extent according to the individual historical optimal position and the population's global optimal position, thus improving the local exploitation ability of the population, but also weakening the global detection ability of the population. A reasonable value of inertia weights can effectively balance the detection and exploitation ability of the population. Generally, in the early stage of population iteration, a larger inertia weight value is chosen to enable the population to detect the solution space effectively; in the later stage of the search, a smaller inertia weight value is chosen to enable the population to quickly perform local optimization search to achieve effective exploitation.

The article "A Model for Analyzing Teaching Quality Data of Sports Faculties Based on Particle Swarm Optimization Neural Network" was published in 2022. Journal: Comput Intell Neurosci.

Both approaches aim to balance the detection and exploitation capabilities of the population and the quality of the searched solutions. This is an education and teaching platform jointly built by teachers and students. A good teaching environment can not only stimulate students' interest in sports learning. Larger inertia weights and scaling factors can improve the population's ability to detect the region of the solution, as shown in Figure 2, and smaller inertia weights and scaling factors can improve the population's ability to exploit the optimal solution in a specific region.

When the neural network hidden unit activation function has no inflection point and is monotonically increasing or monotonically decreasing, when the minimum value of the function is at both ends of the definition domain, then the network with low input-output sensitivity is near both ends of the definition domain. When the neural network hidden unit activation function has an inflection point, the activation function first-order derivative minimum is at both ends of the definition domain or the inflection point according to the discussion of Case 3 and Case 4 above. Therefore, the network with low input-output sensitivity is near the ends or inflection points of the definition domain.

The data preprocessing stage focuses on the initial processing and collation of the raw collected data. The original data is collected from multiple data sources, which appears to be disorganized and contains certain missing, noisy, and inconsistent data, so that it is impossible to directly carry out data mining work, so the researcher needs to process the original data before carrying out data mining work and convert the original disorganized data into normative data that meets the requirements of data mining. The training time of ELM based on heuristic optimization is roughly the same. Although the number of hidden units in the network constructed by these algorithms is small, the time overhead is higher than that of traditional ELM. It mainly contains three processes: data cleaning, data clustering, and data conversion.

For noise filtering, we use data relevance to supplement the missing data, so that the data has a certain degree of integrity; data clustering is mainly to aggregate and categorizes data collected from different data sources to improve the efficiency of data mining; data conversion is mainly to process the categorized data again, following the selected data mining. Data conversion is mainly to reprocess the categorized data and convert it into the data format required by the data mining algorithm following the data requirements of the selected data mining algorithm, to lay the foundation for the data mining work.

The article "A Model for Analyzing Teaching Quality Data of Sports Faculties Based on Particle Swarm Optimization Neural Network" was published in 2022. Journal: Comput Intell Neurosci.

When implementing this link, first, we need to clarify the data itself, according to the data characteristics and application scenarios to choose the appropriate data mining algorithms, such as clustering, regression, association rules, and decision trees. Secondly, based on the algorithm for data mining, and in the process of continuous adjustment of data, finally generate a corresponding model in the data.

### 3.2. Teaching Quality Data Analysis Model Design of Sports Faculties

In the teaching process, the elements that can influence students' learning activities are multiple, both internal and external factors [20]. The external factors are mainly teaching methods and the teaching environment. And the internal factors mainly involve students' learning ability, learning interest, and motivation. Through the analysis of literature, this paper interprets the student factor to mean the specific performance of students' influence on the quality of physical education teaching in teaching activities. It mainly includes students' learning interests and motivation as well as learning ability.

The basic form of realizing private undergraduate education is classroom teaching, and classroom teaching is the driving force to achieve reform and innovation development. The evaluation of classroom teaching quality is to evaluate teachers' classroom teaching ability and urge them to continuously improve their teaching ability to ensure that students get good learning results. The purpose of public physical education classroom teaching quality evaluation refers to the goals and requirements to be achieved by physical education classroom education quality evaluation activities, and the behavior of teaching quality assessment activities can be standardized throughout the process of physical education classroom teaching quality evaluation practice. So, the purpose of teaching quality evaluation must be clarified before implementing public. When evaluating teaching quality in public physical education classrooms, it should be clear why the evaluation should be conducted.

(7) $$\begin{array}{c} X_{\text{new}}=\frac{x+\min\left(X\right)}{\max\left(X\right)+\min\left(X\right)}\times 100\%. \end{array}$$

From Figure 3, it can be seen that 77 people (81.05% of the total) think that the purpose of public classroom is to provide a basis for teachers' appointment, promotion, reward, and punishment, ranking first in the purpose of physical education classroom teaching quality evaluation; 59 people (62.10% of the total) think that the purpose of evaluation is to promote teachers' improvement in teaching, ranking second. The hybrid optimization algorithm based on the improved PSO algorithm not only uses the gradient information of the loss function to ensure the convergence speed of the algorithm, but also maintains the global search ability of the PSO algorithm particle swarm cooperative search. The third place was occupied by 55 people (57.89% of the total) who thought that the purpose of teaching in public physical education classes was in the fourth place and was occupied by 51 people (53.68% of the total) who thought that the purpose of evaluating the quality of teaching in public physical education classes was to optimize school management; the fourth place was occupied by 43 people (45% of the total) who thought that the purpose of evaluating the quality of teaching in public physical education classes was to provide a basis for teachers' training and further training. The fifth place is occupied by 43 students, accounting for 45.26% of the total number of students [21]. The purpose of public physical education classroom teaching quality evaluation is mainly a motivational tool for schools to promote teachers' classroom teaching, and through the feedback of evaluation, teachers can correct their shortcomings in time, promote the continuous improvement of teachers' teaching quality, and realize teachers' personal development, but at this stage, the purpose of public is mostly linked to titles and promotions and fails to evaluate from the purpose of improving teachers' teaching quality and promoting teachers' development.

68.20% of students evaluate the teaching quality of public physical education classrooms because of school regulations [21]. Most colleges and universities link students' final grades with teaching quality evaluation, and students will not be able to check their final grades if they do not evaluate their teaching, so students simply and quickly evaluate their teaching to cope with school requirements, and the results of evaluation do not reflect the real level of teachers. Students do not have a clear understanding.

The article "A Model for Analyzing Teaching Quality Data of Sports Faculties Based on Particle Swarm Optimization Neural Network" was published in 2022. Journal: Comput Intell Neurosci.

From the above three theoretical bases, the principles of physical education, unilaterally evaluating the teaching quality of physical education classroom from students' learning effect, teachers' teaching effect, or teaching environment is one-sided, and the evaluation of physical education classroom teaching quality should be a collection of the above three, also considering teaching. The influence of the teaching environment on the quality of teaching is also considered, and one of the three is indispensable, as shown in Figure 4.

Physical education is an active and lagging subject, and for students, although it is necessary to exert student's initiative in physical education classes and to bring out their physical activities by their habits and behaviors, it is not possible to completely let students play freely. In the construction of informatization, relevant departments of colleges and universities collect and summarize various information and data resources through advanced network and database technology and analyze and process these resources. The formation of physical movement skills is a long-term, step-by-step process, and teachers must play a guiding role in the process of students' physical education learning, for which the teacher's teaching style, verbal behavior, and adequacy of preparation before class are all elements of teaching quality evaluation, forming a warm, harmonious, and cohesive class, so that students can form a correct exercise behavior style and a lifelong exercise ideology.

## 4. Analysis of the Results

### 4.1. Particle Swarm Optimization Neural Network Performance Test Results

In Figure 5, all ELMs optimized based on the heuristic optimization algorithm ((E-ELM, PSO-ELM, IPSO-ELM, and PSOIOS-ELM) trained feedforward networks to have a much smaller number of hidden units than those trained by the conventional ELM, but they take in screening the optimal of the network input layer weights and hidden cell thresholds, and iterations are required. The input-output sensitivity of the single-hidden-layer feedforward network constructed by algorithm PSOIOS-ELM is lower than that of the networks constructed by all algorithms except the algorithm E-ELM. The single-hidden-layer feedforward network constructed by algorithm PSOIOS-ELM has the lowest conditional value of the hidden-layer output matrix, which indicates that the constructed network has good conditional performance, and likewise the network has the highest stability.

The input and output sensitivities of the three PSO-based ELM-constructed networks are similar and much smaller than those of the neural networks constructed by the conventional ELM and E-ELM. They are unable to pass the make-up exam or retake the exam before graduation, which will ultimately affect their normal graduation. The informatization management of colleges and universities can use the existing data for analysis, to take precautions before problems occur. The conditional performance of the networks constructed by algorithms E-ELM, IPSO-ELM, and PSOIOS-ELM is better than that of the conventional ELM and PSO-ELM. The 2 parameters in algorithm PSOIOS-ELM are lower than those in ELM and PSO-ELM and slightly higher than those in algorithms E-ELM and IPSO-ELM 2-parametric values. The training times of ELMs based on heuristic optimization are roughly similar, although these algorithms construct networks with a smaller number of hidden units, but with a higher time overhead than traditional ELMs, all of which are better than the networks constructed by traditional ELM, but all of which are inferior to the networks constructed by algorithm E-ELM. The time overheads of the four evolutionary optimization algorithm-based ELMs are similar but much higher than those of the traditional ELM, with those of the algorithm PSOIOS-ELM slightly lower than those of the other three evolutionary ELMs. In terms of classification performance, PSOIOS-ELM algorithm has the highest test accuracy, as shown in Figure 6.

The article "A Model for Analyzing Teaching Quality Data of Sports Faculties Based on Particle Swarm Optimization Neural Network" was published in 2022. Journal: Comput Intell Neurosci.

From the figure, the test RMSE tends to increase with the increase of tolerance coefficient when approximating the SinC function; on the baseline data classification problem, the test accuracy tends to decrease with the increase of tolerance coefficient. The potential value hidden in the data has not been excavated, the data resources have not been effectively used, and the administrators have no way to find every student with problems that are left alone and provid guiding suggestions for every student with academic problems. As the tolerance factor increases, the input-output sensitivity of the network tends to increase for both the function approximation problem and the basic classification problem. From the figure, the tolerance factor of 0.02 is a reasonable choice in the experiments in this chapter. This experiment provides a reference for the selection of the tolerance coefficient value.

### 4.2. Model Performance Analysis

The secondary school education classroom is teaching quality evaluation index system, and we should uphold a scientific and rigorous attitude to research and adhere to the principle of scientific in organizing and thinking about the literature, that is, the screening of assessment indicators. This has become a research topic and an opportunity for colleges and universities, that is, how to use artificial intelligence technology to tap the potential value hidden in big data to guide teaching decision-making, improve teaching quality, and optimize teachers' teaching behavior. Regardless of which aspect of the research is conducted, the existing teaching quality evaluation system should not be analyzed and considered alone but should be viewed from the perspective of development, based on the existing research results and the main existing evaluation problems to make reasonable judgments, combining teaching elements, students' characteristics, and selecting teaching quality evaluation indicators from various aspects and perspectives, so that the external and internal links can be made. Make the constructed index system carry out comprehensive analysis and integrated evaluation, as shown in Figure 7.

The article "A Model for Analyzing Teaching Quality Data of Sports Faculties Based on Particle Swarm Optimization Neural Network" was published in 2022. Journal: Comput Intell Neurosci.

It shows that the data have a present degree of differentiation. In terms of data dispersion, the standard deviation of most of the measured variable indicators is less than 1, which shows that the data are relatively concentrated. In determining whether a set of data conforms to the normal-terrestrial distribution, it can generally indicate that the data conforms to the normal-terrestrial distribution.

Feedback on learning is a part of feedback theory in education, which is mainly for evaluating the quality of students' learning, and as a part of teaching quality evaluation. The evaluation of students' learning quality does not only refer to the teacher's judgment of students' learning effect, but also the students' evaluation of the learning effect in the classroom, their learning in the physical education classroom, and their evaluation of the teaching style and teaching behavior of the teacher in this class. As educated people, students' physical education learning performance determines to a certain extent how effective the physical education teachers' teaching is. On the other hand, too many hidden units will affect the conditional performance of the network, thereby affecting the stability of the network. Therefore, students' timely teaching feedback, including their evaluation of teachers, can help students' physical education knowledge and motor skills learning, while teachers can improve their teaching style and teaching behaviors based on students' evaluation, which makes the quality of physical education classroom teaching improved, as shown in Figure 8.

Validity is used to examine the extent to which a measurement instrument can correctly measure the traits that need to be measured. Often used is a content validity that is also known as face validity, which refers to the fit and conformity between the measurement target and the measurement content. The questionnaire is evaluated by the researcher or an expert in the field to determine whether the content of the questionnaire meets the purpose and requirements of the measurement. The main influencing factors were attitude toward teaching, verbal ability, ability to demonstrate actions, ability to observe and understand students, and ability to regulate teaching activities. However, putting the teacher-student relationship into the teacher factor (C2) is not very reasonable in theory, so it cannot be used only as an indicator to measure teacher factor.

The article "A Model for Analyzing Teaching Quality Data of Sports Faculties Based on Particle Swarm Optimization Neural Network" was published in 2022. Journal: Comput Intell Neurosci.

Although the indicators of physical education environment measurement were grouped under other dimensions in the factor analysis, theoretically, the physical education environment to a certain extent governs the teaching process. A smaller inertia weight value reduces the impact of the previous generation speed of the particle on the current particle speed, which means that the particle adjusts its flight direction to a large extent according to the individual historical optimal position and the global optimal position of the population, thereby improving the population. For the loss function optimization scenario in convolutional neural networks, the hybrid optimization algorithm is proposed by combining the features of group cooperative search in the improved PSO with the gradient information of the loss function of convolutional neural networks.

## 5. Conclusion

Compared with the gradient learning-based feedforward network learning algorithm, randomly setting the input layer weights and hidden unit thresholds of the network may limit its further performance improvement, mainly because the randomization of the network parameters requires more hidden-layer units, which increases the complexity of the network and limits the improvement of the network generalization performance. When the parameters of the randomized network are nonoptimal or non-near-optimal, the output layer weights calculated by generalized inverse are also nonoptimal or non-near-optimal, which eventually leads to the nonoptimal or non-near-optimal performance of the network. In this study, the weight values of the indicators at each level were obtained by applying the hierarchical analysis method with the results of expert ratings. The weight values of the three-level indicators of teacher teaching behavior, student learning behavior, and teaching environment relative to the quality of secondary school physical education classroom teaching were 0.106, 0.634, and 0.260, respectively, which showed that the student learning behavior dimension had the highest weight value in the evaluation of secondary school physical education classroom teaching quality, followed by teaching environment and finally teacher behavior. The training samples for the experiments are preprocessed GTSRB datasets. The weight parameters of the convolutional neural network were optimized by constructing an improved high-dimensional PSO algorithm combined with the SGD algorithm, ADAM algorithm, and ADAGRAD algorithm, respectively. The final experimental structure reflects that the effect of the hybrid algorithm gains significantly on the SGD algorithm and ADAGRAD algorithm, while the gain effect in the ADAM algorithm is only reflected in the first iteration.

The article "A Model for Analyzing Teaching Quality Data of Sports Faculties Based on Particle Swarm Optimization Neural Network" was published in 2022. Journal: Comput Intell Neurosci.

## Figures and Tables

**Figure 1:** Flowchart of basic PSO.

**Figure 2:** Educational data mining process.

**Figure 3:** Statistics on the awareness of the purpose of public physical education classroom teaching quality evaluation.

**Figure 4:** Comparison of continuity values for each cluster.

**Figure 5:** Corresponding output results when the algorithm PSOIOS-ELM approximates the SinC function.

**Figure 6:** Input-output sensitivity curves of single-hidden-layer stochastic feedforward neural networks trained by ELM on different datasets.

**Figure 7:** Statistical results.

**Figure 8:** Relationship curve between the number of hidden units and test precision.

## Data Availability

The data used to support the findings of this study are available from the author upon request.
